RETRACTED

# Clinical Value Analysis of High-Frequency Ultrasound Combined with Carpal Dorsiflexion Electrophysiological Detection in the Diagnosis of Early Carpal Tunnel Syndrome

**DOI:** 10.1155/2022/6443013

**Published:** 2022-03-29

**Authors:** Yadong Gu, Fei Lu, Shuo Cui, Huafei Zhao, Zhengjiang Yuan

**Affiliations:** Henan Institute of Microsurgery, The First Affiliated Hospital, and College of Clinical Medicine of Henan University of Science and Technology, Luoyang, 471003, China

## Abstract

**Objective:**

To investigate the clinical value of ultrasound combined with electrophysiological examination in the diagnosis of early carpal tunnel syndrome, we aimed to provide a new EMG (electromyography) method for detecting early carpal tunnel syndrome by exploring the wrist back stretch position and electrophysiological examination.

**Methods:**

For the 82-lateral wrist (case group) of 62 patients with clinical symptoms or confirmed carpal tunnel syndrome and 40 normal healthy patients, neuroelectrophysiological measurements were performed using a Keypoint6.0 EMG evoked potentiometer, measuring each group twice: conventional position (before compression) and dorsal wrist extension position. The measures for each measurement included DSL, DML, and CAMP. Measure sensory conduction first and then measure motor conduction. The measurements were analyzed in a comprehensive comparative analysis. Combined ultrasound examination, the positive rate of combined ultrasound examination and electrophysiological examination was compared, respectively.

**Results:**

In the carpal tunnel syndrome (CTS) group, the anterior and posterior median nerve DSL was (4.27 ± 0.73) ms and (4.82 ± 0.65) ms, and SNAP was (13.32 ± 13.68) UV and (12.19 ± 11.04) UV; the median nerve (wrist-bunions) DML was (5.29 ± 1.26) ms and (5.54 ± 1.29) ms, and CMAP was (6.44 ± 2.40) mV and (6.21 ± 2.46) mV. Mid-median DSL and DM in the CTS group L were significantly longer than before compression; median nerve SNAP and CMAP were significantly reduced compared with before compression.

**Conclusion:**

Electrophysiological testing at the dorsal carpal extension position has high diagnostic value in the diagnosis of mild carpal tunnel syndrome. It helps to improve the diagnostic rate of early carpal tunnel syndrome, while providing a more accurate and effective EMG detection of early carpal tunnel syndrome, and combination examination of neuroelectrophysiology and ultrasound can improve the diagnosis rate of compression peripheral nerve diseases and clarify the site, nature, and scope of compression lesions, which is worthy of clinical application.

## 1. Introduction

Middle and ulnar nerve compression is the most common. Electrophysiological examination is the test used to evaluate heart's electrical system and to check for abnormal heart rhythms, which is the current effective means [1]. However, it contains the early existence of many false negatives. More than 40% of the typical carpal tunnel syndrome tests had no abnormalities [2]. The electrophysiology room of our hospital conducted the early diagnosis of carpal tunnel syndrome combined with second lumbrical-interosseus distal motor latency (2LI-DML) to improve the detection rate. However, it cannot provide the neuromorphological changes and the cause of stuck compression [3–5]. Carpal tunnel syndrome (CTS) refers to the clinical symptoms of the median nerve and its branch compression through the bone fiber pipeline under the transverse ligament of the wrist in the hand. It is the most common neurocompression disease in clinical practice, commonly known as “mouse hand” [6]. In 1950, the Phalen reported a large number of CTS cases and gave the first detailed description of the etiology, diagnosis, and treatment of CTS. The patient was diagnosed by the clinician [7]. However, due to the different diagnostic standards and testing methods, the real incidence rate cannot be accurately obtained. The incidence rate is reported abroad as 2.76/100,000, which is better developed in middle-aged women [8]. In recent years, the occurrence of the disease has an obvious younger trend, which may be greatly related to the long-term handicraft work of young patients. The pathogenesis of CTS is still not completely clear, including mechanical compression theory, local microvascular ischemia theory, and vibration theory [9]. Clinically, it mainly relies on clinical symptoms and auxiliary examination for the diagnosis of the disease, according to the severity of the patient nonsurgical treatment or surgical treatment [10–11].

RETRACTED

The carpal tunnel is a hard and inelastic bone structure, whose volume is relatively fixed and is normally filled with tendons and nerves. Any factor that causes the absolute or relatively small size of the carpal tunnel can directly or indirectly compress the median nerve and its branches, causing symptoms. The causes are various, but more than 93% of the causes can be clear [12]. For the treatment of carpal tunnel syndrome, nonsurgical treatment was adopted based on the severity of patient severity [13]. For patients with early CTS, patients who do not be willing to accept surgery, and patients with surgical contraindications due to systemic conditions, conservative treatment is adopted: wrist support therapy, carpal tunnel local injection of corticosteroid hormone or oral neuronutrition drugs, exercise therapy, acupuncture, yoga and oral steroids, and nonsteroid anti-inflammatory drugs. Patients with ineffective conservative treatment, clear carpal tunnel compression, long course of disease, and even muscle atrophy will need surgical treatment. In the traditional surgical plan, cutting the wrist transverse ligament is correct; the middle nerves were subjected to decompression and hydrolysis [14]. Endoscopic carpal tunnel hydrolysis (ECTR) has been gradually applied for CTS [15], which has no damage to the normal tissue on the surface of the median nerve during surgery [16]. In recent years, ultrasonography with the use of high-frequency transducers is confined as a valuable diagnostic tool both for assessing patient eligibility for surgical treatment of CTS and in postoperative assessment of the treatment efficacy. The diagnostic accuracy of high-resolution ultrasound in screening for carpal tunnel syndrome and grading its severity is moderated by age [17].

Since CTS is a compression neurological disease, it is not clear whether EMG sensitivity to CTS can be improved by measuring nerve conduction velocity at the time of median nerve compression [18]. Therefore, this study is aimed at observing the influence of carpal dorsiflexion position on nerve conduction in CTS patients. The clinical application value of ultrasound combined with electrophysiological examination in the diagnosis of early carpal tunnel syndrome provides an intuitive, simple, and accurate electromyographic examination method for carpal tunnel syndrome, improves the diagnosis rate of early CTS, and then provides health guidance for CTS patients to avoid the further development of the disease.

## 2. Materials and Methods

### 2.1. Subject Investigated

The study subjects selected 62 cases of suspected carpal tunnel syndrome or related symptoms from October 2019 to October 2021, 82 side wrist, with an average course of 3 years and 7 months. The clinical case group was collected as the CTS group (experimental group) with inclusion criteria: one or more of the following clinical symptoms: ① three radial sides of the palm of the half finger (thumb, finger, middle finger, ring radial half) numbness, abnormal feeling, or pain; ② median nerve is numb in the dominant area of the palm; ③ night numbness or hand swelling in the morning; ④ numbness increased and shaking; and ⑤ bunion on the palm muscle decline and big fish muscle atrophy. Exclusion criteria were as follows: rheumatoid arthritis, acrohypertrophy, amyloidosis, connective tissue disease, familial disease, hyperparathyroidism, hypothyroidism, tumors, chronic renal failure, cervical spondylosis, congenital carpal tunnel abnormalities, or trauma. The inclusion criteria of the control group were as follows: ① volunteers over 18 years and ② an informed consent form must be signed. This study has been approved by the ethical committee of Henan Institute of Microsurgery.

RETRACTED

### 2.2. Research Technique

Clinical patients (CTS) and normal and healthy people (controls) were measured at the same room temperature (18-25°C), checked using a Keypoint6.0 EMG evoked potentiometer (Vidi, Shenzhen, China), with two measurements, the first measurement (conventional position) and the second measurement [19]. All examinations were performed by the same experienced EMG testing physician. The first measurement was as follows: routine measurement, the patient's upper limb flat put, wrist flat put, relax your palms, and stretch them out. The second measurement was as follows(carpal dorsiflexion 90°, position after finger compression): carpal dorsiflexion 90°, bilateral elbow flexion, forearm pronation, double carpal dorsiflexion, palm relatively close to carpal dorsiflexion 90°, maintain carpal dorsiflexion 90° position 30 seconds later, start measuring again, and hold the position until the end of measurement.

### 2.3. Neuroelectrophysiological Examination

Key point 8-channel EMG/induced potentiometer was used for detection. Nerve conduction examination was performed using the Dantic Key Point EMG machine in the EMG room of our hospital, and patients who were clinically assessed as having idiopathic CTS were examined. The operator was an experienced neuroelectrophysiological technician who was not aware of our clinical findings: Distal motor latency of the median nerve and ulnar nerve, distal motor latency of the median wrist nerve, compound muscle action potential (CMAP), median and ulnar nerve loosening load velocity, sensory nerve velocity (SCV), sensory latent, and sensory nerve action potential (SNAP) amplitude. To examine the median nerve, it has the forearm supine, the elbow straight, the wrist in a neutral position, the palm facing upward, and the fingers straight. To examine ulnar nerve motor conduction, bend the patient's elbow to 90° and take sensory conduction in the same position as median nerve examination. The ulnar nerve conduction examination was performed to exclude peripheral neuropathy with median nerve injury.

① Traditional electrophysiological examination was as follows: sensory motor conduction velocity, amplitude, and latency of median and ulnar nerves; ② second lumbrical and interossei distal motor latency difference (2LI-DML) was used to measure the latency of the second lumbrical and interossei distal motor latency difference and compare the difference; ③ short segment conduction time (SSCT) stimulates the upper and lower parts of the elbow every 1 cm and records the latency and amplitude of CMAP (Figure 1).

RETRACTED

### 2.4. High-Frequency Ultrasound Examination

GE LOGIQ E9 color sonograph with probe frequency 6-15MHZ.Cross-section area (cross-sectional area, CSA). Philips IU22 color Doppler ultrasound diagnostic instrument and linear array probe were used. During the examination, the subject takes a sitting position with the forearm, wrist, and palm horizontally placed and palm upward. High-frequency probe was used to carry out cross-section (especially cross-section continuous sliding scanning method) and longitudinal and sequential scanning on the metacarpal side, dorsal side, and internal and external side of the wrist of the patient (Figures 2(a) and 2(b)).

### 2.5. Electrophysiological Standards

① The latency period, amplitude, and conduction velocity of the distal sensorimotor of median and ulnar nerves were determined by dang Jingxia's EMG Diagnosis and Clinical Application in 2020 [13]: NCV (nerve conduction velocity) slowness at the entrapment > 10 m/s. The amplitude of the two action potentials decreased >50%; ② 2LI-DML was as follows: motor latency of median nerve and distal ulnar nerve >0.4 ms; ③ SSCT: the latency difference between two points is ≥ 0.6 ms.

### 2.6. Ultrasound Standard

Unilateral lesions with a healthy arm nerve as a control were as follows: bilateral lesion reference (20): carpal tunnel syndrome: CSA 10.4 mm^2^; and elbowed tunnel syndrome: CSA 7.5 mm^2^.

### 2.7. Statistical Analysis

The collected data collected were analyzed by mean standard deviation (*x* ± *s*) and SPSS25.0 statistical software for statistical analysis. After checking data for normal distribution and variance homogeneity, continuous data were compared using multiple Student *t*-tests or two-way ANOVA. After the median and ulnar compression, all *P* values are two-tailed, and *P* values <0.05 are considered significant (^∗^*P* < 0.05, ^∗∗^*P* < 0.01, and ^∗∗∗^*P* < 0.001). The data are represented as mean ± S.E.M. or the median with 10 and 90 percentiles.

## 3. Result

### 3.1. Comparative Analysis of the General Data between the CTS and Control Groups

Carpal tunnel syndrome (CTS group)was as follows: 62, 25 males, 37 females, 82 lateral wrists, mean age of 52.27 years (31-72 years), normal healthy individuals (control), 40, 24 females, 16 males, 80 lateral wrists, and mean age of 52.69. There was no significant difference between age and sex (*P* > 0.05) (Table 1).

### 3.2. Measurement Results before and after Median Nerve and Ulnar Nerve Compression in the CTS Group

In the CTS group, the sensory conduction terminal latency (DSL) of the anterior and posterior median nerve was (4.27 ± 0.73) ms and (4.82 ± 0.65) ms, which was a significant difference between the two, and the latency after compression was greater than before compression, with a statistically significant comparison between the two groups (*P* < 0.05) (Table 2).

RETRACTED

Mild CTS is defined as sensory distal latency of >3.4 ms and< 3.9 ms and peak sensory latency of >4.6 ms and Motor distal latency ≤ 4.5 ms. And mild-severe CTS is defined as sensory distal latency > 3.9 ms and< 5.6 ms and peak sensory latency > 6.1 ms, and motor distal latency <4.9 ms. In this study, SNAP was (13.32 ± 13.68) UV and (12.19 ± 11.04) UV. There was a significant difference between the two groups. The amplitude of wave after compression was lower than that before compression and significantly decreased, with statistical significance between the two groups (*P* < 0.05) (Table 3).

The motor conduction terminal latency (DML) of the anterior and posterior median nerve (wrist-bunion muscle) was (5.29 ± 1.26) ms, (5.54 ± 1.29) ms, which can see that the incubation period after compression was greater than before compression and significantly prolonged, which was statistically significant between the two groups (*P* < 0.05). The combined muscle action potentials (CMAP) of anterior and posterior median nerves (carpal-Abducus hallucis brevis) were (6.44 ± 2.40) mV and (6.21 ± 2.46) mV. The amplitude of wave after compression was significantly lower than that before compression, with statistical significance between the two groups (*P* < 0.05) (Table 4).

### 3.3. Comparison of Electrophysiological and Ultrasound Examination Results of Typical Cases

There were 62 cases of carpal tunnel and cubital tunnel syndrome (bilateral 18 cases, unilateral 44 cases) and 46 cases of traditional electrophysiological examination abnormal (abnormal rate 74.19%). Median nerve 2Li-DML abnormalities were found in 49 (62, 79.03%). There were 27 abnormal ulnar nerve SSCT (32 in total, the abnormal rate was 84.38%). There were combined electrophysiological examination (traditional and 2LI-DML, SSCT examination) abnormal 54 cases (abnormal rate 87.09%). There were 55 cases with abnormal ultrasound alone (88.70%) and 58 cases with abnormal electrophysiological ultrasound (93.54%). There was statistically significant difference in the positive rate between combined electrophysiological examination and traditional electrophysiological examination (*P* < 0.01), and there was statistically significant difference between electrophysiological examination combined with ultrasound examination and combined electrophysiological examination (*P* < 0.01) (Table 5).

RETRACTED

### 3.4. Comparison of Traditional Electrophysiology, Combined Electrophysiology, and Electrophysiology Combined with Ultrasound Results in Atypical Cases

There are 2 carpal tunnel and cubital tunnel syndromes (bilateral 8 cases, unilateral 26 cases) and traditional electrophysiological examination abnormal 25 cases (abnormal rate 59.52%). Median nerve 2Li-DML was abnormal in 20 cases (26 cases, abnormal rate 76.92%). Ulnar nerve SSCT was detected in 13 sides (a total of 16 sides, abnormal rate 81.25%). Combined with electrophysiological (traditional and 2LIDML, SSCT examination) abnormality of 37 sides (abnormality rate 88.10%), there were 34 cases with abnormal ultrasound alone (abnormal rate 80.95%) and 39 cases with abnormal electrophysiological ultrasound combined (abnormal rate 92.86%). The positive rate of combined electrophysiological examination was significantly different from traditional electrophysiological examination (*P* < 0.01). The positive rate of electrophysiological examination combined with ultrasonography was significantly different from that of electrophysiological examination (*P* < 0.01) (Table 6).

## 4. Discussion

Carpal tunnel syndrome is one of the most common diseases of all peripheral neurotonic disorders. The incidence was only 0.6% in men, compared with 5.8% in women [21]. The disease is especially common in middle-aged and elderly women and is presumed to be related to long-term family manual labor and altered premenopausal and postmenopausal sex hormone levels [22]. The carpal tunnel is a relatively fixed, inelastic rigid bone pipe, this narrow bone pipeline with nine tendons and its tendon sheath and the median nerve passes through, and any factor that can reduce carpal tunnel volume or relatively more content will squeeze the median nerve and cause carpal tunnel syndrome. Oliveira et al. [23] found that the patient first felt numbness or pain in the three fingers of the radius, holding weakness, with the middle finger, and the heaviest symptoms at night or in the morning, appropriate symptoms of shaking the wrist can be reduced, and wrist Tinel and Phalen signs are positive. Kerasnoudis et al. [24] found that big fish between electromyography and wrist refers to the median nerve conduction speed determination of nerve damage; although electrophysiological diagnosis is a special diagnostic standard of wrist syndrome, but it cannot provide necessary help for surgery, cannot look directly around the median nerve, high-frequency ultrasound can well show the median nerve and wrist tendon and is conducive to find the cyst, schwannoma, lipoma, hematoma, and other causes of carpal tunnel syndrome [25].

Ultrasound showed thickening of median nerve membrane, thickening of diameter, enhancement of echo, uneven internal echo, interruption of linear parallel echo, and unclear boundary [26]. The direct evidence of ultrasonic diagnosis of carpal tunnel syndrome was swelling and thickening of median nerve. Studies have shown that the cross-sectional area of the upper median nerve of the carpal tunnel >0.09 cm^2^ can be used as a reliable diagnostic standard. In this study, carpal tunnel syndrome caused by the thickening of the transverse carpal ligament was selected to observe the thickness of the transverse carpal ligament and the corresponding changes of the median nerve [27]. In carpal tunnel syndrome, the carpal tunnel is poorly defined and deformed, and there may be extensive adhesions to its internal structures. The area values of the patients in this group were all >0.09 cm^2^. Gao et al. [28] reported that the median nerve was most easily displayed at the level of the pea bone (the proximal carpal tunnel) with the largest cross-sectional area. It should be noted that the probe should be operated perpendicular to the median nerve. In addition, the operation should not be too hard; otherwise, the compression of the probe will cause deformation of the median nerve. High-frequency ultrasound can be dynamic imaging, time-saving, and low cost; relative to electrophysiological examination, painless; can also clearly show the median nerve and surrounding adjacent structures; and evaluate the surgical effect by comparing the median nerve before and after the operation.

RETRACTED

Zuniga et al. [29] has shown that when severe hallux short abductor muscle atrophy of CTS is serious, conventional method cannot be recorded on thumb short abductor muscle action potentials, and severe patients with routine inspection may not be feeling action potential; in this case, it is difficult to determine the parts of the median nerve injury, and the second loop shape muscle often associated with the lighter. Therefore, this technique can be used to record the difference in latency between the action potential and the median nerve-ulnar nerve. Thumb short abductor muscle and the second loop muscle at the same time dominated by the median nerve, muscle between the bones, swayed by ulnar nerve in the wrist control thumb short abductor muscle fibers than dominate the second loop shape muscle shallower; so, the wrist median nerve damage to dominate thumb short abductor muscle of nerve fiber damage is more serious, in the thumb short abductor muscle action potential and is lesser. It is a better method to record potential. Since the interosseous muscle is located below the second lumbrical muscle, the two can share a recording electrode, thus avoiding the influence of exogenous factors (temperature, stimulation, spacing of recording points, et al.). Usually, the recording electrode was placed about 1 cm lateral to the midpoint of the third metacarpal bone (the second lumbricus-interosseous muscle surface projection), the reference electrode was located on the surface of the distal phalanx of the index finger, and the stimulation electrode was located at the median or ulnar nerve body surface projection of the wrist, 12 cm away from the recording electrode. In the normal population, the latency difference between the two was less than 0.4 ms, and when the latency difference was greater than 0.4 ms, the median nerve injury was indicated. Moran et al. [30] diagnosed median nerve injury by comparing median nerve-second lumbrical muscle DML with ulnar nerve-interosseous muscle DML. Subsequent studies by Babaei-Ghazani et al. [31] showed that the second lumbric-interosseous technique had high sensitivity in the diagnosis of CTS, even in mild CTS where abnormalities could not be detected by conventional techniques. Mohammadi et al. [32] in China further studied the detection of different degrees of CTS by the second lumbric-interosseous muscle technique, and the results showed that this technique can be used to detect various degrees of CTS, especially for severe CTS with a diagnostic sensitivity of 86.7%, which has significant diagnostic significance for severe CTS accompanied by multiple neuropathy. Mohammadi et al. [33] have shown that the second lumbric-interosseous technique has the highest sensitivity compared to other techniques in the diagnosis of severe CTS with polyneuropathy.

RETRACTED

Electrophysiology is the gold standard for diagnosing CTS but does not show neural architecture [34]. High-frequency ultrasound can clearly show the internal neural structure. This study shows that the combined examination can improve the diagnostic rate of peripheral nerve compression diseases, be more intuitive to anatomical variation and occupation, clarify the site, nature, and scope of the lesion, and provide a reliable basis for preoperative and postoperative evaluation and dynamic review.

## 5. Conclusion

This study shows that electrophysiological testing at the dorsal carpal extension position has high diagnostic value in the diagnosis of mild carpal tunnel syndrome. It helps to improve the diagnostic rate of early carpal tunnel syndrome, while providing a more accurate and effective EMG detection of early carpal tunnel syndrome, and combination examination of neuroelectrophysiology and ultrasound can improve the diagnosis rate of compression peripheral nerve diseases and clarify the site, nature, and scope of compression lesions, which is worthy of clinical application.

RETRACTED

## Figures and Tables

**Figure 1:** (a, b) Median nerve sensory conduction examination.

**Figure 2:** (a, b) High-frequency ultrasound images of carpal tunnel syndrome. The cross-section of carpal tunnel and median nerve [1] was observed and recorded, and the tissues around tendon [2] and tendon sheath [3], synovium [4], and articular cartilage [5] were observed.

**Table 1:** Comparative analysis of the general data between the CTS and control groups.

Group	Gender (man/female)	Age (year)
CTS group	25 : 37	52.27 ± 14.39
Control group	2 : 3	52.69 ± 13.62
*P*	>0.05	>0.05

**Table 2:** Data values of the parameters before and after median nerve compression in the CTS.

CTS group	Nervi medians			
	DSL (ms)	SNAP (UV)	DML (ms)	CMAP (mV)
Before oppression	4.27 ± 0.73	13.32 ± 13.68	5.29 ± 1.26	6.44 ± 2.40
After oppression	4.82 ± 0.65	12.19 ± 11.04	5.54 ± 1.29	6.21 ± 2.46
*P*	< 0.05	< 0.05	< 0.05	< 0.05

**Table 3:** Data values for the parameters before and after median nerve compression between clinical typing in the CTS group.

CTS group	Nervi medianus			
	DSL (ms)	SNAP (UV)	DML (ms)	CMAP (mV)
Mild group				
Before oppression	4.17 ± 0.63	13.56 ± 12.68	5.25 ± 1.22	6.69 ± 2.51
After oppression	4.73 ± 0.54	13.09 ± 11.07	5.51 ± 1.27	6.27 ± 2.48
*P*	< 0.05	< 0.05	< 0.05	< 0.05
Middle-severe group				
Before oppression	4.38 ± 0.87	13.28 ± 11.73	5.31 ± 1.29	6.32 ± 2.39
After oppression	4.86 ± 0.65	13.24 ± 11.59	5.34 ± 1.26	6.30 ± 2.42
*P*	< 0.05	< 0.05	< 0.05	< 0.05

**Table 4:** Data values of the parameters before and after ulnar nerve compression in the CTS group.

CTS group	Ulnar nerve			
	DSL (ms)	SNAP (UV)	DML (ms)	CMAP (mV)
Before oppression	2.19 ± 0.27	19.31 ± 10.99	2.23 ± 0.40	14.33 ± 3.69
After oppression	2.22 ± 0.21	19.26 ± 11.02	2.24 ± 0.26	14.28 ± 3.48
*P*	>0.05	>0.05	>0.05	>0.05

**Table 5:** Comparison of different diagnostic methods in typical cases.

Group	Traditional electrophysiology	Combined electrophysiology	Electrophysiology was combined with ultrasound
(+)	56	54	58
(-)	26	8	4
*t*		22.242	43.909
*P*		<0.001	<0.001

**Table 6:** Comparison of different diagnostic methods in atypical cases.

Group	Traditional electrophysiology	Combined electrophysiology	Electrophysiology was combined with ultrasound
(+)	25	37	39
(-)	17	5	3
*t*		8.347	23.908
*P*		0.002	0.001

## Data Availability

The data used to support this study is available from the corresponding author upon request.
